# Effects of Multimodal Analgesia Combined with Auricular Point Therapy on Physical and Mental Stress and Rehabilitation Quality of Patients with Meniscus Injury during the Perioperative Period

**DOI:** 10.1155/2022/3130956

**Published:** 2022-08-17

**Authors:** Yuanyuan Yao, Guiyang Yu, Jianbo Lu, Tian Han, Huizhen He

**Affiliations:** Second Central Hospital of Baoding, Baoding 072750, China

## Abstract

**Objective:**

To investigate the effect of multimodal analgesia combined with auricular point therapy on physical and mental stress and rehabilitation quality of patients with meniscus injury during the perioperative period.

**Methods:**

148 patients in our hospital from October 2019 to October 2021 who were scheduled to undergo meniscus surgery were selected and grouped according to the order of file establishment, with 74 cases in each. The control group was given routine analgesia, and the observation group was given multimodal analgesia combined with auricular point therapy. The pain level (visual analogue scale (VAS)), physical and mental stress (heart rate (HR), mean arterial pressure (MAP), depression scale (PHQ-9), and anxiety scale (GAD-7)), complications, rehabilitation quality, and analgesia satisfaction were observed.

**Results:**

The VAS scores of pain in the observation group were lower than those in the control group at 6 hours before operation and at 6 hours, 24 hours, and 72 hours after operation (*P* < 0.05). The MAP, HR, PHQ-9, and GAD-7 scores of the observation group were lower than those of the control group 6 hours before operation (*P* < 0.05). There was no significant difference in MAP, HR, PHQ-9, and GAD-7 scores between the two groups at 6 hours and 24 hours after operation (*P* > 0.05). The analgesic satisfaction of the observation group was better than that of the control group (*P* < 0.05). The incidence of complications in the observation group was 8.11% compared with 12.16% in the control group, which was not statistically significant (*P* > 0.05). The first exhaust, getting out of bed, and hospital stay in the observation group were shorter than those in the control group (*P* < 0.05).

**Conclusion:**

Multimodal analgesia combined with auricular acupuncture therapy is effective in perioperative patients with meniscus injury. It can reduce perioperative pain, reduce physical and mental stress, and promote early postoperative recovery through a variety of analgesic mechanisms.

## 1. Introduction

Meniscus injury is a common injury disease of the knee joint. At present, surgery is an important way to restore the integrity and stability of the meniscus, which can effectively reduce the symptoms of pain, swelling, and joint locking [1]. However, perioperative and early postoperative rehabilitation exercise pain is an important factor that leads to severe physical and mental stress and affects the compliance and rehabilitation quality of postoperative rehabilitation training. Therefore, it is very important to strengthen perioperative analgesia and management for postoperative joint function recovery.

Multimode analgesia is a kind of analgesic program that combines the application of drugs with different methods or mechanisms to make them have synergistic effects, so as to reduce the dosage of analgesics and improve the analgesic effect, and has achieved remarkable effects in clinical application [2]. In recent years, in addition to drug analgesia, it has been reported that auricular point pressing bean as a nondrug intervention can reduce the dosage of early postoperative analgesics by stimulating the auricle acupoints, without vomiting, nausea, and other adverse reactions [3]. Therefore, this study combined multimode analgesia and auricular acupoint therapy for perioperative patients with meniscus injury surgery, comprehensively analyzed the physical and mental stress, rehabilitation quality, and pain degree, in order to provide new ideas for improving the rehabilitation quality of patients.

## 2. Materials and Methods

### 2.1. Patient Information

From October 2019 to October 2021, 148 patients undergoing meniscus surgery in our hospital were selected. There were no differences between the two groups in gender, age, inducing factors, course of disease, scope of surgical resection, and history of knee joint (*P* > 0.05), as shown in Table 1. This study was approved by the hospital ethics committee.

### 2.2. Patient Selection Criteria

Inclusion criteria include the following: arthroscopy, confirmed meniscus injury combined with clinical symptoms and signs; treated with arthroscopic surgery; clear language expression and consciousness; and signed the informed consent. Exclusion criteria include the following: cognitive dysfunction; people allergic to analgesic drugs; and patients with acute or chronic serious diseases.

### 2.3. Intervention Method

The control group took routine analgesia:

1. Preoperative: no analgesic drugs were used.
2. Postoperative: parecoxib 40 mg was given orally, once every 12 h, for 3 d. On the 1st postoperative day, 200 mg celecoxib was given orally, twice a day, and tramadol 1co was given orally, 3 times a day for 7 d. If the patient still felt unbearable pain, 100 mg tramadol was injected intramuscular depending on the situation.

The observation group received multimode analgesia combined with auricular acupoint therapy:

(1) Multimode analgesia:
  (1.1) 48 hours before surgery: 200 mg celecoxib capsules were taken orally, once every 12 hours, and physical analgesia therapy such as relaxation therapy was informed; night 20 : 00, take a comfortable lying position, close the eyes, focus on the body, relax, and contract head-trunk-upper extremity-buttocks-lower extremity-feet successively. After the muscles of the whole body are completely relaxed, imagine a beautiful, calm, natural scene, feel happy time with your family, have hope for the future, and achieve the purpose of relaxation. Or music therapy, according to the patient's personal characteristics and personality, provide personalized music repertoire, extroverts, soft, and soothing music, and introvert, mainly to positive music. The volume should be tolerated by patients.
  (1.2) Before skin excision: 40 mg parecoxib injection intravenously
  (1.3) Immediately after the surgery: intravenous controlled analgesia was taken, 2 *μ*g/kg sufentanil injection and 50 mg flurbiprofen ester injection were dissolved in 150 mL normal saline at 2 mL/h, the pressure was 0.5 mL, the shortest interval was 15 min, and ice bag cold compress was continued around the incision for 24 hours.
  (1.4) 10 hours after surgery: before homotomy
  (1.5) 2–7 d after surgery: same as 48 hours before surgery
(2) Auricular point therapy: since the start to the end of the 7 d after admission, concrete steps as follows: lateral auricular portal nerve, large nerve points, subcortical, small pillow nerve, and sympathetic, such as acupuncture and alcohol disinfection. The adhesive tape (0.6 cm × 0.6 cm) with the seeds of cowherb seed was applied to the auricular acupoint, and then, a little pressure was applied until the patient appeared sore and numb, 3–5 times per day.

### 2.4. Observation and Evaluation

1. Pain degree: visual analogue scale (VAS) [4] was used to evaluate the changes of pain at admission, 6 hours before surgery, 6 hours, 24 hours, and 72 hours after surgery. The score ranged from 0 to 10. The higher the score, the more severe the pain. The scale had good reliability and validity in pain assessment of patients with meniscus injury, and the consistency Cronbach's *α* coefficient was 0.865.
2. Physical and mental stress: heart rate (HR) and mean arterial pressure (MAP) were recorded at admission, 6 hours before surgery, and 6 hours and 24 hours after surgery, respectively, and psychological stress state was assessed by patient health questionnaire depression scale (PHQ-9) [5] and generalized anxiety scale (GAD-7) [6]. The total score of the former was 0–27, and the higher the score, the more severe the depression. The latter score was 0–20, and the higher the score was, the more serious the anxiety was. Cronbach's *α* coefficient of consistency of the above scale was 0.812 and 0.869, respectively.
3. Analgesia satisfaction: based on expert opinions and previous literature [7], the satisfaction was divided into 3 grades according to VAS score: satisfactory VAS score <3, general VAS score 3–5, and unsatisfactory VAS score >5.
4. Complications: these include joint popping, sensation of falling apart, and joint effusion.
5. Rehabilitation quality: the first exhaust, out of bed activity, and hospital stay in the two groups were counted.

### 2.5. Statistical Analysis

SPSS 23.0 software was used and measurement data (±*s*) were expressed. The homogenous *t*-test of variance was performed for data conforming to normal distribution, while the *t-*test was used for heterogeneity of variance. The *χ*^2^ test was used for counting data *n* (%). Ridit analysis and *U* test were used for grade data. *P* < 0.05 meant the difference was statistically significant.

## 3. Results

### 3.1. Comparison of the Pain Degree of the Two Groups

On admission, there was no significant difference in VAS score between the two groups (*P* > 0.05). VAS scores of the observation group were lower than those of the control group at 6 hours before surgery as well as 6 hours, 24 hours, and 72 hours after surgery, and the differences were statistically significant (*P* < 0.05). The results are shown in Table 2 and Figure 1.

### 3.2. Comparison of the Physical and Mental Stress Indicators in Two Groups

There were no significant differences in MAP, HR, PHQ-9, and GAD-7 scores between the two groups on admission (*P* > 0.05). MAP, HR, PHQ-9, and GAD-7 scores in the observation group were lower than those in the control group at 6 hours before operation (*P* < 0.05). Besides, there were no significant differences in MAP, HR, PHQ-9, and GAD-7 scores between the two groups at 6 hours and 24 hours after surgery (*P* > 0.05). The results are shown in Table 3 and Figure 2.

### 3.3. Comparison of the Analgesic Satisfaction in Two Groups

After evaluation, the analgesic satisfaction in the observation group was better than that in the control group, and the difference was statistically significant (*P* < 0.05), as shown in Table 4.

### 3.4. Comparison of the Complications in Two Groups

The complication rate of 8.11% in the observation group was not significantly different from 12.16% in the control group (*P* > 0.05), as shown in Table 5.

### 3.5. Comparison of Rehabilitation Quality in the Two Groups

The first exhaust, get out of bed time, and hospital stay in the observation group had shorter than the control group, and the differences were statistically significant (*P* < 0.05), as shown in Table 6.

## 4. Discussion

At present, arthroscopy is the main method to treat meniscus injury. However, studies have reported that perioperative pain is closely related to the rehabilitation process and prognosis for patients with limb injury [8]. At the same time, studies have confirmed that after arthroscopic surgery, active rehabilitation training is one of the important determinants of the final outcome [9]. Therefore, strengthening perioperative analgesia management, reducing pain degree, alleviating patients' physical and mental stress response, and promoting early postoperative functional exercise are of great importance for postoperative rehabilitation and prognosis.

Multimode analgesia is the combination of drugs or methods with different analgesic mechanisms to complement each other in order to enhance analgesia synergism and reduce the dosage of analgesic drugs. Studies have found that multimode analgesia can not only improve the analgesic effect but also reduce the side effects of anesthesia to maximize the effect/side effects ratio, so as to achieve balanced analgesia [10]. In recent years, multimode analgesia has been clinically considered as an ideal analgesic method in the perioperative period, which can effectively shorten the length of hospital stay and reduce the adverse reactions such as vomiting and nausea caused by anesthesia, and is favored by the majority of doctors and patients. In view of this, this study applied it to the perioperative analgesic management of patients with meniscus injury. In order to further strengthen the analgesic effect and reduce the physical and mental stress caused by pain and surgery, this study combined with the traditional Chinese medicine treatment of auricular acupoint pressing beans, sticking the medicine beans on the auricular acupoint through adhesive tape for moderate stimulation, so as to achieve the purpose of external treatment. Traditional Chinese medicine believes that auricular points are related to the physiological functions corresponding to human meridians. A large number of studies have confirmed that auricular acupoint stimulation can produce double stimulation to the cerebral cortex, such as excitation and inhibition, and then exert analgesic and immune regulation effects [11, 12]. In addition, studies have reported that auricular acupoint therapy can reduce the dosage of postoperative analgesic drugs without occurrence of anesthesia-related adverse reactions [13].

This study combined multimode analgesia with auricular acupoint therapy. The results showed that the VAS score of the observation group was lower than that of the control group at 6 hours before surgery and at different time points after surgery, and the analgesic satisfaction was better than that of the control group (*P* < 0.05). Therefore, the combined plan adopted in this study had a significant analgesic effect and was widely recognized and satisfied by patients. In addition, from the perspective of stress, stress refers to the nonspecific stress state generated by stress factors in the body when the body is subjected to intense damage stimulus including physiological and psychological parts, namely, physical and mental stress [14]. Psychological stress is an important factor that affects patients' attitude towards care and causes intense physical stress, while abnormal physiological changes can reduce immunity and aggravate inflammatory response, which is not conducive to postoperative recovery [15]. Therefore, this study based on patients with physical and mental stress monitoring found that MAP, HR, PHQ-9, and GAD-7 scores in the observation group at 6 hours before surgery were lower than that of the control group (*P* < 0.05). These indicated that multimodal analgesia combined with auricular application therapy could decrease the degree of physical and mental stress through reducing the preoperative pain, showing that the blood pressure, HR, and anxiety depression were decreased. However, this study showed that there were no significant differences in MAP, HR, PHQ-9, and GAD-7 scores between the two groups at 6 hours and 24 hours after surgery (*P* > 0.05). The reason is that analgesia management was adopted in both groups after surgery. Although the observation group had better analgesia, the pain degree in both the groups was lower, and the effect on physical and mental stress was relatively small.

Studies have reported that the pain caused by surgical injurious stimulation and the disease itself can cause neuroendocrine stress response, resulting in excessive metabolism such as elevated blood glucose and water and sodium retention, which hinder postoperative recovery of patients [16]. Affected by pain stimulation, most patients reject early postoperative ambulation, which affects rehabilitation training compliance and is not conducive to prognosis [17]. This study for the first time found that the first exhaust, get out of bed time, and hospital stay in the observation group were shorter than that of the control group (*P* < 0.05), indicating that multimodal analgesia combined with auricular application therapy could achieve good analgesia effect through a variety of analgesic effect mechanism and reduce the adverse effects of traumatic stimulation on patients' body and mind. In addition, patients with pain relief can get out of bed as early as possible, which plays an irreplaceable role in promoting early postoperative recovery and shortening hospital stay [2]. However, this study showed that there was no statistical significance in the incidence of postoperative complications between the two groups (*P* > 0.05), suggesting that in addition to strengthening the analgesic effect, complications prevention and management should be done to further reduce the risk of complications in clinical.

In conclusion, multimode analgesia combined with auricular acupoint therapy has a significant effect on perioperative patients with meniscus injury, which can relieve perioperative pain, reduce physical and mental stress, and promote early postoperative recovery through various analgesic mechanisms. However, there are some shortcomings in this study such as limited sample size and single-center study, so multicenter and large-sample study should be adopted in the future to explore the application effect of this research scheme in a more comprehensive and systematic way.

## Figures and Tables

**Figure 1:** Changes in pain trends.

**Figure 2:** Changes in physical and mental stress.

**Table 1:** Comparison of general data.

Project	Observation group (*n* = 74)	Control group (*n* = 74)	*t*/*χ*^*2*^	*P*
Male/female	40/34	38/36	0.108	0.742
Age (year)	38.96 ± 9.10	41.02 ± 10.36	1.285	0.201
Disease duration (months)	3.25 ± 1.12	2.98 ± 1.03	1.526	0.129
Predisposing factors			0.449	0.799
Long-term weight squat	36 (48.65)	32 (43.24)		
Knee sprain	24 (32.43)	26 (35.14)		
Knee osteoarthritis	14 (18.92)	16 (21.62)		
Surgical resection			0.668	0.414
Half cut	68 (91.89)	65 (87.84)		
Full cut	6 (8.11)	9 (12.16)		
History of the knee			0.363	0.547
Yes	7 (9.46)	5 (6.76)		
No	67 (90.54)	69 (93.24)		

**Table 2:** Comparison of pain degree between two groups (±*s*, points).

Group	*n*	On admission	6 hours before surgery	6 hours after surgery	24 hours after surgery	72 hours after surgery
Observation group	74	5.20 ± 2.33	5.12 ± 2.10	2.18 ± 0.56 act	2.74 ± 0.58	2.10 ± 0.54
Control group	74	5.48 ± 1.97	3.24 ± 1.56	2.46 ± 0.63	3.10 ± 0.47	2.68 ± 0.48
*t*		0.789	6.182	2.858	4.148	6.906
*P*		0.431	<0.001	0.005	<0.001	<0.001

**Table 3:** Comparison of psychological stress between two groups (±*s*, points).

Time	Group	*n*	MAP	HR	PHQ-9	GAD-7
On admission	Observation group	74	118.24 ± 10.87	124.25 ± 12.47	7.74 ± 3.01	9.22 ± 1.28
	Control group	74	121.36 ± 13.58	122.48 ± 11.20	8.18 ± 2.69	8.78 ± 1.20
	*t*		1.543	0.125	0.938	1.102
	*P*		0.125	0.246	0.350	0.315
6 hours before surgery	Observation group	74	92.36 ± 8.10	96.47 ± 10.35	5.10 ± 2.11	6.24 ± 1.98
	Control group	74	116.78 ± 10.47	114.74 ± 9.54	7.25 ± 1.85	8.35 ± 2.01
	*t*		15.869	11.165	6.591	10.857
	*P*		<0.001	<0.001	<0.001	<0.001
6 hours after surgery	Observation group	74	89.58 ± 5.69	82.36 ± 6.75	3.89 ± 1.65	4.01 ± 1.47
	Control group	74	91.01 ± 7.54	83.58 ± 5.98	4.24 ± 1.78	4.21 ± 1.69
	*t*		0.896	1.164	1.241	0.768
	*P*		0.412	0.246	0.217	0.444
24 hours after surgery	Observation group	74	84.74 ± 6.10	81.44 ± 5.63	2.01 ± 0.85	2.78 ± 0.62
	Control group	74	86.55 ± 7.54	83.10 ± 6.85	2.13 ± 1.02	2.98 ± 0.96
	*t*		1.605	1.611	1.234	1.506
	*P*		0.111	0.109	0.324	0.134

**Table 4:** Comparison of analgesic satisfaction between two groups (%).

Group	*n*	Satisfied	General	Dissatisfied
Observation group	74	57 (77.03)	16 (21.62)	1 (1.35)
Control group	74	43 (58.11)	18 (24.32)	13 (17.57)
*u*		2.359		
*P*		0.018		

**Table 5:** Comparison of complications between two groups (%).

Group	*n*	Knuckle snapping	Joint loss	Joint effusion	Incidence
Observation group	74	2 (2.70)	3 (4.05)	1 (1.35)	6 (8.11)
Control group	74	3 (4.05)	4 (5.41)	2 (2.70)	9 (12.16)
*χ* ^2^					0.668
*P*					0.414

**Table 6:** Comparison of rehabilitation quality between two groups (±*s*, d).

Group	*n*	First exhaust time	Get out of bed time	Hospital stay
Observation group	74	0.89 ± 0.25	1.48 ± 0.56	6.75 ± 2.11
Control group	74	1.36 ± 0.35	1.97 ± 0.74	8.97 ± 2.89
*t*		9.400	4.542	5.337
*P*		<0.001	<0.001	<0.001

## Data Availability

The labeled datasets used to support the findings of this study are available from the corresponding author upon request.
